The article "Analysis and Study on Epidemiological Features and Prognosis of Nephrotic Syndrome in Xinjiang and Heilongjiang" was published in 2021. Journal: Comput Math Methods Med.

# Analysis and Study on Epidemiological Features and Prognosis of Nephrotic Syndrome in Xinjiang and Heilongjiang

**DOI:** 10.1155/2021/8802670

**Published:** 2021-11-24

**Authors:** Jizhang Liu, Yuxia Zhong, Liangduan Ding, Ayinuer Tuluhong, Burebi Maihemuti, Tianxiong Pan, Mingjie Wu, Hailong Chen, Chen Lu

**Affiliations:** ^1^Nephrology, Daqing Oilfield General Hospital, Daqing City, Heilongjiang Province 163000, China; ^2^Nephrology, People's Hospital of Shache County, Kashgar, Xinjiang Uygur Autonomous Region 844700, China; ^3^Nephrology, The First Affiliated Hospital of Xinjiang Medical University, Xinjiang Uygur Autonomous Region 930011, China

## Abstract

**Backgrounds:**

The pathogenesis of nephrotic syndrome (NS) is complex, and there are differences between regions. This study attempted to collect clinicopathological data of patients diagnosed with NS in Xinjiang and Heilongjiang in the past 2 years, so as to explore the onset features of NS and treatment and prognosis of patients in the two regions.

**Methods:**

Clinical data of 375 patients diagnosed with NS using renal biopsy in Xinjiang and Heilongjiang from March 2019 to March 2021 were collected. Clinical data of patients before treatment were collected, and the chi-square test was utilized to compare the differences in the sex distribution of two groups. The *U* test was utilized to compare abnormal distribution continuous data between two groups, such as age, hemoglobin, plasma albumin, proteinuria, and triglycerides. Independent sample *t*-test was utilized to compare normal distribution continuous data between two groups, such as serum total protein, serum creatinine, blood urea nitrogen, glomerular filtration rate, and total cholesterol. The independent sample *t*-test was also used to compare the immunoglobulin levels and complement levels between the two groups after treatment, including IgA, IgG, IgM, C3, and C4. Kaplan-Meier method was used to analyze and plot the cumulative curves of complete remission rate and partial remission rate.

**Results:**

For 275 NS patients from Xinjiang, the male-to-female ratio was 0.81 : 1. For 84 patients from Heilongjiang, the male-to-female ratio was 1.05 : 1. The onset ages of patients in Xinjiang and Heilongjiang were 22-45 years old and 22-47 years old, respectively. Respectively, there were 221 cases (80.36%) and 66 cases (78.57%) of primary NS in Xinjiang and Heilongjiang. There were 54 cases (19.64%) and 18 cases (21.43%) of secondary NS in Xinjiang and Heilongjiang, respectively. There was no statistically significant difference in cause distribution between the two regions (*p* = 0.756). After treatment, immunoglobulin levels (IgA (*p* = 0.009), IgG (*p* = 0.002), IgM (*p* < 0.001)) and complement C3 (*p* < 0.001) and C4 (*p* < 0.001) levels in Xinjiang and Heilongjiang were statistically significant. 129 cases in Xinjiang (46.91%) and 55 cases in Heilongjiang (65.48%) were treated with glucocorticoid (GC) combined with immunosuppressive therapy, respectively. After receiving treatment, 67 (24.36%) of 275 patients in Xinjiang achieved complete remission, 166 (60.36%) achieved partial remission, 22 (26.19%) of 84 patients in Heilongjiang achieved complete remission, and 56 (66.67%) achieved partial remission, and there was no statistically significant difference in remission rate between the two regions (*p* = 0.159). Patients in Xinjiang and Heilongjiang achieved complete remission at an average of 10.34 weeks (9.98-10.70) and 9.95 weeks (9.26-10.65), respectively. There was no significant difference in complete remission rates between the two regions (*p* = 0.663). Patients in Xinjiang and Heilongjiang achieved partial remission at an average of 8.76 weeks (8.38-9.14) and 7.99 weeks (7.33-8.65), respectively. There was no significant difference in the partial remission rate between the two regions (*p* = 0.065).

The article "Analysis and Study on Epidemiological Features and Prognosis of Nephrotic Syndrome in Xinjiang and Heilongjiang" was published in 2021. Journal: Comput Math Methods Med.

**Conclusion:**

The causes of NS in Xinjiang and Heilongjiang were similar. After treatment, there were differences in immunoglobulin levels (IgA, IgG, IgM) and complement levels (C3, C4) in the two regions. The main treatment methods used in the two regions were GC combined with immunosuppressive therapy. The prognosis of patients in the two regions was similar. The complete remission rate and partial remission rate after treatment in the two regions were similar, and the average time required to achieve complete remission and partial remission was also similar.

## 1. Introduction

Nephrotic syndrome (NS) is a nonspecific nephropathy and characterized by large amount of proteinuria, hypoalbuminemia, hyperlipidemia, and peripheral edema [1]. The pathogenesis of primary NS has not yet been fully elucidated. Patients with primary NS often have varying complications, which can be life-threatening if improperly treated [2]. Studies have demonstrated that factors like environment [3], public health conditions [4], race, and gene [5] may affect the onset of nephropathy. NS can be caused by primary nephropathy or multiple secondary causes [2]. Generally, main pathotypes of primary NS include minimal change disease (MCD), membranous nephropathy, focal segmental glomerulosclerosis (FSGS), and IgA nephropathy (IgAN). Besides, main secondary NS includes Henoch-Schönlein purpura nephritis (HSPN), lupus nephropathy (LN), and diabetic nephropathy [6]. There are various pathotypes of NS, and treatment for each pathotype is different. Additionally, patients' response to those treatments and their prognoses are also greatly different. Hence, the identification and diagnosis of NS should be highly valued. However, previous studies showed that the pathotypes of NS vary in races, ages, and regions. For instance, a study on NS patients in Japan by Sugiyama et al. [7] indicated that the top three pathotypes of NS are MCD (45.7%), membranous nephropathy (35.6%), and FSGS (11.3%). Additionally, a study by Schena demonstrated that membranous nephropathy (32.9%), FSGS (12.3%), and MCD (12.0%) are the commonest pathotypes of NS patients in Italy [8]. For age classification, a study on 1,523 Chinese NS patients exhibited that MCD (33.0%), LN (23.0%), idiopathic membranous nephropathy (IMN) (37.9%), and IMN (42.3%) [9] are the commonest causes in NS patients aged 14-24, 25-44, 45-59, and ≥60 years, respectively. Hence, NS pathotypes vary in races, ages, and regions, and understanding the pathological spectrum of NS is of great significance for its treatment and clinical practice.

The article "Analysis and Study on Epidemiological Features and Prognosis of Nephrotic Syndrome in Xinjiang and Heilongjiang" was published in 2021. Journal: Comput Math Methods Med.

Respectively, Xinjiang and Heilongjiang are on the westernmost and easternmost borders of China. These two regions showed great differences in residential areas and ethnics composition. Statistically, people of ethnic minorities accounts for 68.4% of total population in Xinjiang in 2018, which is remarkably higher than those in Heilongjiang (5.26%). Besides, in Xinjiang, rural permanent resident population is 12.14 million (48%), which is dramatically higher than 10.95 million (34%) in Heilongjiang [10]. Furthermore, it was reported that residential areas and economic conditions are the independent correlation factors of kidney damage. For example, in rural areas, economic development independently correlates with proteinuria [10]. Our study is aimed at analyzing the epidemiological feature, pathological spectrum, and prognosis of NS patients in Xinjiang and Heilongjiang. Our efforts may bring insight to the prevention, diagnosis, and treatment of nephropathy in two regions, so as to improve patients' prognosis.

## 2. Materials and Methods

### 2.1. Data Collection

Patients who were diagnosed with NS in Heilongjiang and Xinjiang from March 2019 to March 2021 were selected. NS was defined as 24-hour urinary protein > 3.5 g/d, plasma albumin < 30 g/L, hyperlipidemia, and edema, among which the first two symptoms were basic standards. Inclusive criteria are as follows: NS patients who were local residentials or who have been settled for at least 5 years in either Xinjiang or Heilongjiang. Exclusive criteria are as follows: NS patients who had incomplete data, undergone renal replacement therapy, or who were pregnant. Clinical data of patients before treatment were collected: sex, age, hemoglobin, plasma albumin, serum total protein, serum creatinine, proteinuria, blood urea nitrogen, glomerular filtration rate, triglycerides, and total cholesterol. Clinical data of patients after treatment were collected: immunoglobulin levels (IgA, IgG, IgM) and complement levels (C3 and C4).

The article "Analysis and Study on Epidemiological Features and Prognosis of Nephrotic Syndrome in Xinjiang and Heilongjiang" was published in 2021. Journal: Comput Math Methods Med.

### 2.2. Therapeutic Schedules [11]

In primary NS, the therapeutic schedule for membranous nephropathy was glucocorticoid (GC) + immunosuppressant and GC + calcineurin inhibitor (CNI); the treatment plan for IgA nephropathy was GC monotherapy or GC + immunosuppressive therapy; minimal change nephropathy was treated with GC monotherapy, GC + immunosuppressive agent, or GC + CNI therapy. Considering the drug resistance and hormone dependence caused by GC monotherapy, patients with secondary NS in both regions were treated with GC + immunosuppressive agents or traditional Chinese medicine. Lupus nephropathy was treated with GC + immunosuppressive agents or GC + CNI therapy.

For GC monotherapy, the initial drug was prednisone 1 mg/(kg∗d), taken orally for 8 weeks, once every other day to reduce hormonal side effects.

For GC + immunosuppressive therapy, immunosuppressive agents exerted a synergistic therapeutic effect in addition to GC therapy, mainly included cyclophosphamide (CTX), 2 mg/(kg∗d), orally once or twice a day, or 200 mg, intravenous injection every other day, withdrawal after 6-8 g accumulation.

Other treatment options included GC + CNI, cyclosporine, and mycophenolate mofetil. GC + traditional Chinese medicine was applied for patients with diabetic nephropathy, hypertensive nephropathy, etc. The dosage of CNI was 0.05-0.10 mg/(kg∗d) of tacrolimus and 3 mg/(kg∗d) of cyclosporine, taken orally on an empty stomach twice, and the dosage was gradually reduced in 2-3 months. Traditional Chinese medicine was mainly tripterygium glycosides, 10-20 mg, orally three times a day.

### 2.3. Evaluation Criteria for Remission and Prognosis of Patients in Two Regions after Treatment [12]

Patients' examination data and clinical information were collected 12 weeks before or after treatment. Complete remission (CR) of NS was defined as proteinuria < 0.3 g/d and the disappearance of other NS symptoms such as edema, hypoproteinemia, and hyperlipidemia. Besides, partial remission (PR) was defined as proteinuria = 0.3-3.5 g/d with a 50% reduction of baseline and a stable level of serum creatinine (SCr). Invalid (NR) was defined as a reduction of proteinuria baseline < 50% or the increase of proteinuria.

### 2.4. Statistical Analysis

Statistical analysis was conducted on SPSS (26.0). Continuous measurement data conforming to Gaussian distribution and uniform variance were subjected to two independent sample *t*-test. Continuous measurement data not conforming to normal distribution were subjected to Mann–Whitney *U* test. The enumeration data were compared by chi-square test for differences between groups, and the Kaplan-Meier method was utilized for survival analysis of remission rate, and *p* < 0.05 was considered statistically significant.

The article "Analysis and Study on Epidemiological Features and Prognosis of Nephrotic Syndrome in Xinjiang and Heilongjiang" was published in 2021. Journal: Comput Math Methods Med.

## 3. Results

### 3.1. Basic Information of Patients in Two Regions before Treatment

As shown in Table 1, there were 275 NS patients from Xinjiang, which included 123 males (44.73%) and 152 females (55.27%) with a male-to-female ratio of 0.81 : 1. Meanwhile, there were 84 NS patients from Heilongjiang, which included 43 males (51.19%) and 41 females (48.81%) with a male-to-female ratio of 1.05 : 1. There was no difference in the ratio of males to females between the two regions (*p* = 0.298). Patients in Xinjiang were 31 years old (22, 45), while those in Heilongjiang were 33 years old (22, 47). The differences in ages of patients in two regions were not statistically significant (*p* = 0.835).

For patients in Xinjiang, the hemoglobin level was 121.70 g/L (103.60, 137.20); the plasma albumin level was 24.27 g/L (19.58, 28.29); the blood total protein level was 59.81 ± 0.75 g/L; the blood creatinine level was 75.26 ± 1.59 *μ*mol/L; proteinuria level was 5.46 g/d (4.53, 6.45); blood urea nitrogen level was 6.23 ± 0.11 mmol/L; glomerular filtration rate level was 70.16 ± 0.93 mL/min; triglyceride level was 2.81 mmol/L (1.67, 4.05); total cholesterol level was 7.85 ± 0.15 mmol/L. For patients in Heilongjiang, the hemoglobin level was 117.12 g/L (111.29, 124.21); the plasma albumin level was 21.75 g/L (18.37, 25.80); the blood total protein level was 55.92 ± 0.33 g/L; the blood creatinine level was 89.61 ± 0.69 *μ*mol/L; proteinuria level was 5.02 g/d (4.19, 5.79); blood urea nitrogen level was 8.00 ± 0.24 mmol/L; glomerular filtration rate level was 63.83 ± 1.36 mL/min; triglyceride level was 3.64 mmol/L (2.75, 4.91); total cholesterol level was 7.03 ± 0.23 mmol/L. Except for hemoglobin level, other levels were different in the two regions (*p* < 0.05).

### 3.2. Differences in Pathological Types, Immunoglobulin, and Complement of NS in Patients from Two Regions

According to the pathogenesis, NS can be classified into primary NS and secondary NS. As demonstrated in Table 2, NS patients in both regions were dominated by primary NS which included 221 cases (80.36%) in Xinjiang and 66 cases (78.57%) in Heilongjiang. Besides, membranous nephropathy was the most common in both regions, which included 81 cases (36.65%) in Xinjiang and 38 cases (57.58%) in Heilongjiang. IgA nephropathy came second, including 46 cases (20.81%) in Xinjiang and 15 cases (22.73%) in Heilongjiang. MCD occurred in 32 (14.48%) xinjiang patients and 5 (7.58%) Heilongjiang patients. Respectively, secondary NS in Xinjiang and Heilongjiang were 54 cases (19.64%) and 18 cases (21.43%). Among the secondary NS, lupus nephropathy was the commonest, including 20 cases (37.04%) in Xinjiang and 5 cases (27.78%) in Heilongjiang. There was no statistical significance in differences in pathological types between NS patients in two regions (*p* = 0.756).

The article "Analysis and Study on Epidemiological Features and Prognosis of Nephrotic Syndrome in Xinjiang and Heilongjiang" was published in 2021. Journal: Comput Math Methods Med.

After treatment, the immunoglobulin and complement levels of patients in Xinjiang and Heilongjiang are presented in Table 3. In patients from Xinjiang, IgA level was 1.73 ± 0.03 g/L; IgG level was 4.91 ± 0.19 g/L; IgM level was 1.58 ± 0.02 g/L; C3 complement level was 1.19 ± 0.01 g/L; C4 complement level was 0.25 ± 0.00 g/L. In patients from Heilongjiang, IgA level was 1.89 ± 0.04 g/L; IgG level was 3.83 ± 0.12 g/L; IgM level was 2.81 ± 0.03 g/L; C3 complement level was 0.99 ± 0.02 g/L; C4 complement level was 0.29 ± 0.01 g/L. There was statistical significance between IgA level (*p* = 0.009), IgG level (*p* = 0.002), IgM level (*p* < 0.001), C3 complement level (*p* < 0.001), and C4 complement level (*p* < 0.001) of patients in the two regions (*p* < 0.05).

### 3.3. Treatments and Prognoses of NS Patients in Two Regions

As demonstrated in Table 4, in Xinjiang, 65 NS patients (23.64%) were treated with GC solely, 129 patients (46.91%) were treated with combination therapy of GC and IS, and 81 patients (29.45%) were treated with other therapeutic approaches. In Heilongjiang, 12 patients (14.29%) were treated with GC solely, 55 patients (65.48%) were treated with combination therapy of GC and IS, and 17 patients (20.24%) were treated with other therapeutic approaches. The differences between two regions were of statistical significance (*p* = 0.011).

As exhibited in Table 4, after NS patients in Xinjiang were treated for 12 weeks, 67 of them (24.36%) attained CR, 166 patients (60.36%) attained PR, and 42 patients (15.27%) attained NR. In Heilongjiang, 22 patients (26.19%) achieved CR, 56 patients achieved PR (66.67%), and 6 patients (7.14%) achieved NR. The differences between two regions were not statistically significant (*p* = 0.159).

As illustrated in Figures 1 and 2, patients in Xinjiang achieved CR at an average of 10.34 weeks (95% CI: 9.98-10.70) and PR at an average of 8.76 weeks (95% CI: 8.38-9.14); patients in Heilongjiang achieved CR at an average of 9.95 weeks (95% CI: 9.26-10.65) and PR at an average of 7.99 weeks (95% CI: 7.33-8.65). There was no significant difference in CR rates (*p* = 0.663) and PR rates (*p* = 0.065) between the two regions.

The article "Analysis and Study on Epidemiological Features and Prognosis of Nephrotic Syndrome in Xinjiang and Heilongjiang" was published in 2021. Journal: Comput Math Methods Med.

## 4. Discussion

As a common clinical syndrome, NS is not an independent disease. NS is a syndrome that is caused by permeability damage of glomerular capillary filtration membrane induced by divergent diseases and factors. Besides, it is also a major cause that results in end-stage renal disease [13].

In different regions and hospitals, male NS patients are generally more than female NS patients because males are more addicted to smoking and drinking and have a higher occurrence rate of hypertension and hyperlipidaemia. A single-center clinical study in Beijing showed that male NS patients (55.6%) are significantly more than female NS patients (44.4%) [9]. Similarly, a study on adult NS patients in Pakistan demonstrated that male NS patients accounts for 63.6%, which is remarkably more than female NS patients who accounts for 36.4% [14]. In our study, the male-to-female ratio of NS patients in Heilongjiang was about 1.05 : 1. Surprisingly, female NS patients in Xinjiang account for 55.27%, which was markedly more than male NS patients who account for 44.73%. Similar to our results, a study on glomerular disease showed that 492 (54.85%) out of 897 patients with glomerular disease in Xinjiang were females [15]. The high-risk group of NS in the two regions was 22-47 years old, indicating that NS is most common in young people, which is consistent with the results of a study from India [16].

In our study, NS in Xinjiang and Heilongjiang was dominated by primary NS which accounts for 80.36% and 78.57% of the total cases, respectively. The primary cause of primary NS in both regions was membranous nephropathy. These data were similar to those reported by Western countries [17] but different from the data reported by other countries [7, 18]. These results may be related to atmospheric pollution. Due to the influence of sandstorm in Xinjiang and coal burning in Heilongjiang, the concentration of PM 2.5 in the environment of the two regions is high. Long-term exposure to high concentrations of PM 2.5 is associated with an increased risk of membranous nephropathy [3, 19]. Hence, the high morbidity of membranous nephropathy in the two regions may be related to air pollution. As for secondary NS, the primary causes in Xinjiang were lupus nephropathy and diabetic nephropathy, while lupus nephropathy and nontypical membranous nephropathy were the primary causes in Heilongjiang. Similar to our results, a single-center epidemiological study of nephropathy in China showed that the most common cause of secondary glomerulonephritis was systemic lupus erythematosus (SLE), accounting for 54.3% [20].

The article "Analysis and Study on Epidemiological Features and Prognosis of Nephrotic Syndrome in Xinjiang and Heilongjiang" was published in 2021. Journal: Comput Math Methods Med.

The main causes of NS proteinuria are the enhancement of glomerular filtration membrane permeability. Besides, urinary protein loss results in a decrease of blood IgG. Previous studies have found that serum immunoglobulin and complement levels in NS patients vary in different stages of the disease and patients with different pathological types. For example, it was reported that there is a remarkable decrease of the serum immunoglobulin IgG, a normality of IgA, and an increase of IgM in active NS patients, compared with the healthy control group. In remission period, the IgG, IgA, and IgM levels of NS patients were observed to be markedly increased compared with those of patients in the corresponding active NS period [21]. In addition, a study compared the concentration of serum immunoglobulin of children with idiopathic minimal-change nephrotic syndrome (INS) and nephrotic syndrome secondary to chronic glomerulonephritis (CGN). This study found that serum immunoglobulin IgG and IgA levels were significantly reduced in patients with INS or CGN nephropathy. Besides, mean serum immunoglobulin IgM concentrations of INS patients were more than twice the normal levels before, during and after successful treatment with steroids. However, serum immunoglobulin IgM was not equivalent increased in patients with CGN [22]. Besides, studies also displayed that the difference in immunoglobulin level may be related to the geographical environment of the patients. The serum immunoglobulin IgG and IgA levels of patients with primary glomerular disease in Xinjiang were significantly higher than the serum immunoglobulin IgG and IgA levels of patients with pediatric primary nephrotic syndrome in Jilin, Northeast China. Meanwhile, the IgM level of patients in Xinjiang was significantly lower than that of patients in Jilin [15, 23], which is consistent with our results. In this study, after the patients received treatment, there were differences in overall immune albumin levels and complement levels in the two regions. The main manifestation was that the average immune albumin IgA level (1.73 g/L) of patients in Xinjiang was lower than that of patients in Heilongjiang (1.89 g/L), indicating that overall treatment and prognosis of patients in Xinjiang were better than those in Heilongjiang after GC combined with immunosuppressive therapy.

At present, the core of clinical treatment for NS is aimed at its main pathological and physiological links, namely, the treatment of large amounts of proteinuria caused by glomerular membrane filter lesions, negative transformation or reduction of proteinuria, and the improvement of plasma albumin. The drugs used for the treatments included GCs such as prednisone and methylprednion, as well as immunosuppressants like cyclophosphamide, cyclosporine plus RAAS blockers, nonsteroidal anti-inflammatory drugs, etc. [24, 25]. These drugs are the main drugs for reducing albuminuria. For membranous nephropathy with a high morbidity, Kidney Disease: Improving Global Outcomes (KDIGO) guidelines suggested that the patients can be treated with primarily cyclophosphamide in combination with corticosteroids for 6 months [26], if the patients meet the criteria for immunosuppressive therapy. A recent multicenter study from the UK showed that patients treated with corticosteroids and nitrobutyric mustard have better renal outcomes than patients treated with corticosteroids plus cyclosporine or supportive therapy [27]. For micropathic nephropathy, corticosteroids are recommended by the KDIGO guidelines to induce the remission of micropathic nephropathy in adults [26]. Hence, Different treatment options should be selected for different NS pathological types. Although there are differences in treatment options between the two regions, Xinjiang and Heilongjiang both utilized the GC + IS therapy. Besides, the results displayed that the difference in CR rate and PR rate between the two regions was not statistically significant, and the prognosis of patients in the two regions was similar.

The article "Analysis and Study on Epidemiological Features and Prognosis of Nephrotic Syndrome in Xinjiang and Heilongjiang" was published in 2021. Journal: Comput Math Methods Med.

Through the analysis and study on the epidemiological features and prognoses of 359 NS patients in Xinjiang and Heilongjiang, we preliminarily obtained the pathological characteristics of NS in the two regions. There are both similarities and differences with the reports of other regions at home and abroad, but our study well reflects the characteristics of the two regions. In general, despite similar prognosis of patients in the two regions, a large sample size of NS patients remains warranted for stratified analysis. Besides, this study only studied the pathological characteristics of adult patients, the choice of treatment options, and the degree of remission and prognosis after treatment. We should also expand the discussion about pediatric patients and compare the onset characteristics of adults and children to guide the medication plan. Our study is expected to play a role in promoting the pathological diagnosis and clinical treatment of NS, and meanwhile, provide reference for prognosis of NS patients.

## Figures and Tables

**Figure 1:** Cumulative curves of complete remission rate based on Kaplan-Meier method.

**Figure 2:** Cumulative curves of partial remission rate based on Kaplan-Meier method.

**Table 1:** Basic information of patients in two regions before treatment.

Item		Xinjiang (*N* = 275)	Heilongjiang (*N* = 84)	*p* value
Sex (%)				0.298
Male		123 (44.73%)	43 (51.19%)	
Female		152 (55.27%)	41 (48.81%)	
Age (years)		31 (22, 45)	33 (22, 47)	0.835
Hemoglobin (g/L)		121.70 (103.60, 137.20)	117.12 (111.29, 124.21)	0.191
Blood albumin (g/L)		24.27 (19.58, 28.29)	21.75 (18.37, 25.80)	0.004
Serum total protein (g/L)		59.81 ± 0.75	55.92 ± 0.33	<0.001
Serum creatinine (*μ*mol/L)		75.26 ± 1.59	89.61 ± 0.69	<0.001
Proteinuria (g/day)		5.46 (4.53, 6.45)	5.02 (4.19, 5.79)	0.001
Blood urea nitrogen (mmol/L)		6.23 ± 0.11	8.00 ± 0.24	<0.001
Glomerular filtration rate (mL/min)		70.16 ± 0.93	63.83 ± 1.36	0.001
Triglyceride (mmol/L)		2.81 (1.67, 4.05)	3.64 (2.75, 4.91)	<0.001
Total cholesterol (mmol/L)		7.85 ± 0.15	7.03 ± 0.23	0.006

The article "Analysis and Study on Epidemiological Features and Prognosis of Nephrotic Syndrome in Xinjiang and Heilongjiang" was published in 2021. Journal: Comput Math Methods Med.

**Table 2:** Pathogenesis classification of NS patients in two regions.

Type of NS		Xinjiang (*N* = 275)	Heilongjiang (*N* = 84)	*p* value^a^
Primary NS		221 (80.36%)	66 (78.57%)	0.756
	Membranous nephropathy	81 (36.65%)	38 (57.58%)	
	IgA nephropathy	46 (20.81%)	15 (22.73%)	
	MCD	32 (14.48%)	5 (7.58%)	
	Mesangial proliferative glomerulonephritis	30 (13.57%)	3 (4.55%)	
	Focal segmental glomerular sclerosis	11 (4.98%)	2 (3.03%)	
	Membranoproliferative glomerulonephritis	5 (2.26%)	1 (1.52%)	
	Endocapillary proliferative glomerulonephritis	13 (5.88%)	1 (1.52%)	
	Crescentic glomerulonephritis	3 (1.36%)	1 (1.52%)	
Secondary NS		54 (19.64%)	18 (21.43%)	
	Hepatitis B-associated nephritis	1 (1.85%)	2 (11.11%)	
	Diabetic nephropathy	9 (16.67%)	2 (11.11%)	
	Lupus nephropathy	20 (37.04%)	5 (27.78%)	
	Purpura nephritis	5 (9.26%)	2 (11.11%)	
	Amyloidosis nephropathy	5 (9.26%)	1 (5.56%)	
	Nontypical membranous nephropathy	4 (7.41%)	3 (16.67%)	
	Hypertension-induced kidney injury	5 (9.26%)	2 (11.11%)	
	ANCA-related tubulointerstitial nephropathy	3 (5.56%)	0 (0.00%)	
	Other	2 (3.70%)	1 (5.56%)	

^a^Primary NS vs. secondary NS.

**Table 3:** Differences in immunocomplexes and complement deposition between NS patients in two regions after treatment.

Types of immunocomplex	Xinjiang (*N* = 275)	Heilongjiang (*N* = 84)	*p* value
IgA (g/L)	1.73 ± 0.03	1.89 ± 0.04	0.009
IgG (g/L)	4.91 ± 0.19	3.83 ± 0.12	0.002
IgM (g/L)	1.58 ± 0.02	2.81 ± 0.03	<0.001
C3 (g/L)	1.19 ± 0.01	0.99 ± 0.02	<0.001
C4 (g/L)	0.25 ± 0.00	0.29 ± 0.01	<0.001

**Table 4:** Treatment and prognosis of NS patients in two regions.

Item	Xinjiang (*N* = 275)	Heilongjiang (*N* = 84)	*p* value
Therapeutic approach			0.011
GC	65 (23.64%)	12 (14.29%)	
GC + IS	129 (46.91%)	55 (65.48%)	
Other	81 (29.45%)	17 (20.24%)	
Prognosis			0.159
CR	67 (24.36%)	22 (26.19%)	
PR	166 (60.36%)	56 (66.67%)	
NR	42 (15.27%)	6 (7.14%)	

The article "Analysis and Study on Epidemiological Features and Prognosis of Nephrotic Syndrome in Xinjiang and Heilongjiang" was published in 2021. Journal: Comput Math Methods Med.

## Data Availability

The data and materials in the current study are available from the corresponding author on reasonable request.
